The article "Delivery of Bioactive Lipids from Composite Microgel-Microsphere Injectable Scaffolds Enhances Stem Cell Recruitment and Skeletal Repair" was published in 2014. Journal: PLoS One.

# Delivery of Bioactive Lipids from Composite Microgel-Microsphere Injectable Scaffolds Enhances Stem Cell Recruitment and Skeletal Repair

**DOI:** 10.1371/journal.pone.0101276

**Published:** 2014-07-31

**Authors:** Anusuya Das, Daniel A. Barker, Tiffany Wang, Cheryl M. Lau, Yong Lin, Edward A. Botchwey

**Affiliations:** 1 Department of Orthopaedic Surgery, University of Virginia, Charlottesville, Virginia, United States of America; 2 Department of Biomedical Engineering, University of Virginia, Charlottesville, Virginia, United States of America; 3 Department of Otolaryngology, University of Virginia, Charlottesville, Virginia, United States of America; 4 Department of Biomedical Engineering, Georgia Institute of Technology, Atlanta, Georgia, United States of America; UNIFESP Federal University of São Paulo, Brazil

## Abstract

In this study, a microgel composed of chitosan and inorganic phosphates was used to deliver poly(lactic-co-glycolic acid) (PLAGA) microspheres loaded with sphingolipid growth factor FTY720 to critical size cranial defects in Sprague Dawley rats. We show that sustained release of FTY720 from injected microspheres used alone or in combination with recombinant human bone morphogenic protein-2 (rhBMP2) improves defect vascularization and bone formation in the presence and absence of rhBMP2 as evaluated by quantitative microCT and histological measurements. Moreover, sustained delivery of FTY720 from PLAGA and local targeting of sphingosine 1-phosphate (S1P) receptors reduces CD45+ inflammatory cell infiltration, promotes endogenous recruitment of CD29+CD90+ bone progenitor cells and enhances the efficacy of rhBMP2 from chitosan microgels. Companion *in vitro* studies suggest that selective activation of sphingosine receptor subtype-3 (S1P_3_) via FTY720 treatment induces smad-1 phosphorylation in bone-marrow stromal cells. Additionally, FTY720 enhances stromal cell-derived factor-1 (SDF-1) mediated chemotaxis of CD90+CD11B-CD45- bone progenitor cells *in vitro* after stimulation with rhBMP2. We believe that use of such small molecule delivery formulations to recruit endogenous bone progenitors may be an attractive alternative to exogenous cell-based therapy.

## Introduction

Injury of bone and supporting vasculature induces a wound healing cascade marked by an initial inflammatory response (complement activation, recruitment of monocytes/macrophages, clearance of damaged tissue) and the subsequent recruitment and differentiation of progenitor cells. Several peptide-based factors such as bone morphogenic protein-2 (BMP-2), vascular endothelial growth factor (VEGF), and fibroblast growth factor (FGF) influence these processes and accelerate bone regeneration. However, many challenges involved with healing critical size defects (CSD) such as the need to accelerate bone formation and enhance defect site vascularization may not be overcome through delivery of growth factors alone, and numerous studies have explored adjunct delivery of exogenous stem and progenitor cell sources [1], [2], [3], [4].

The article "Delivery of Bioactive Lipids from Composite Microgel-Microsphere Injectable Scaffolds Enhances Stem Cell Recruitment and Skeletal Repair" was published in 2014. Journal: PLoS One.

Mesenchymal stem cells (MSCs) in particular have been investigated extensively as potential therapeutic agents for treating CSDs [2], [5], [6]. MSCs release a multitude of cytokines, and can differentiate into osteoblasts *in vivo*, and many studies have shown that co-administration of bone marrow derived mesenchymal stem cells (BMSCs) and osteoinductive factors such as BMP-2 accelerates the process of cranial defect healing [2], [7]. However, many studies also suggest that use of exogenous cells may be limited by poor engraftment and poor differentiation *in vivo* [8]. A possible alternative to the use of exogenous cells in this context is the local delivery of sphingolipid growth factors such as sphingosine 1-phosphate (S1P) to promote formation of new blood vessels and induce recruitment of host stem and progenitor cells from the vessel networks and surrounding tissues [9], [10]. Enhancing endogenous stem cell contributions to bone repair through the use novel small molecules to increase their recruitment to the injury site via enhanced defect site vascularization and migration may provide a safe and cost effective alternative to conventional exogenous cell-based therapy [11], [12], [13].

S1P is pleiotropic, autocrine- and paracrine-signaling sphingolipid that is released into the blood upon platelet activation. It binds to a family of five high affinity G-coupled receptors (S1P_1_–S1P_5_) to direct a wide range of biological processes triggered during endogenous bone wound healing, including stimulating osteoblast migration [14], and promoting mature cell survival [10], [15]. Harnessing S1P receptor signaling to enhance bone regeneration can be accomplished by using selective pharmacological agonists and/or antagonists of specific S1P receptors [16], [17], [18]. FTY720, an agonist at receptors S1P_1_, S1P_3–5_, has a systemic half-life of 20 hours [19] and is physiologically more stable compared to native S1P ligand (half life  = 2 hours [20]), or BMP-2 (half life  = 16 min [21]) for clinical applications.

In this study, a vehicle based on chitosan and inorganic phosphates was used to deliver FTY720 to a critical size cranial defect animal model. The effect of FTY720 on the migration of BMSCs was evaluated through transwell migration assays and flow cytometry. We show that in addition to local inflammation resolution [22] and enhanced vascularization [16], [17], [18], FTY720 may aid in bone regeneration by increasing the migration of circulating BMSCs towards the injury site. The selected vehicle formulation is particularly attractive due to the chitosan's ability to solidify at body temperature, a phenomenon known as thermogelling [23], which imparts ease of delivery to the bone defect site. BMP-2 loaded-chitosan gel was infused with FTY720-loaded PLAGA microspheres and injected as per previous studies [2] to encourage vascularization and bone healing. The current CSD study in Sprague Dawley rats compared the effects of dual delivery of FTY720 and BMP-2 on bone healing to those of either FTY720 or BMP-2 alone. The dosage of BMP-2 used was equivalent to the dose previously shown to result in defect healing when combined with an external source of mesenchymal stem cells [2]. Here, we examine the effect of enhancing endogenous progenitor cell recruitment via increased vascularization and enhancement of SDF-1/CXCR4 mediated chemotaxis of progenitor cells in an effort to validate a cell-free strategy for increasing progenitor cell content at a site of bone injury. Bone growth in the defect was evaluated bi-weekly using microCT, vascularization was measured at the end of 9 weeks via Microfil-enhanced imaging, and local inflammatory response/progenitor cell recruitment was evaluated with immunohistochemistry.

The article "Delivery of Bioactive Lipids from Composite Microgel-Microsphere Injectable Scaffolds Enhances Stem Cell Recruitment and Skeletal Repair" was published in 2014. Journal: PLoS One.

## Materials and Methods

### 2.1 Transwell Migration Assays

Bone marrow cells were collected from the tibia of Sprague Dawley rats (Charles River), and serum starved for 2 hours. The cell suspension of 2 million cells/ml was pre-treated with serum free media (SFM), 10 ng/ml BMP-2 (ProspecBio, East Brunswick, NJ, USA), 10 ng/ml FTY720 (Cayman Chemical, Ann Arbor, MI, USA) or both for 30 min and then re-suspended in serum free DMEM (Invitrogen Life Technologies, Carlsbad, CA, USA). 100 µl of the pre-treated cell suspension was added to the top well of 5 µm transwell inserts (Costar) in a 24-well plate. The bottom of the wells contained 600 µl of serum free DMEM alone, or serum free DMEM with 12.5 nM SDF-1 (ProspecBio) or serum free DMEM with 12.5 nM S1P (Cayman Chemical). The different pretreated cells were allowed to migrate towards each of the different solutions at the bottom of the transwells for 4 hours at 37°C, and then the number of cells at the top and the bottom of the transwell membrane were counted using an automatic cell counter.

### 2.2 Flow Cytometry

Whole bone marrow was isolated from C57Bl/6 mice, and was treated with FTY720, BMP-2 or both for 1 hour after 1 hour of serum starvation. MSCs were gated for using CD90 (eBiosciences, San Diego, CA, USA), CD29 (eBiosciences), and Sca-1 (Biolegend, San Diego, CA, USA), and the amount of smad-1 and phosphorylated smad-1 (Cell Signaling Technologies, Beverly, MA, USA) was quantified as percent positive cells over total cells. Flow cytometry was performed according to standard procedures and was analyzed on a FACS Aria II cell sorter (BD, Franklin Lakes, NJ, USA).

The article "Delivery of Bioactive Lipids from Composite Microgel-Microsphere Injectable Scaffolds Enhances Stem Cell Recruitment and Skeletal Repair" was published in 2014. Journal: PLoS One.

The cells that migrated towards SDF-1 in the migration assay were collected from the bottom of the transwells and treated with monoclonal antibodies to CD45 (Biolegend), CD11b (Biolegend) and CD90 (eBioscience) prior to flow cytometry performed according to standard procedures on a 9 color CyAn flow cytometer (Beckman Coulter, Brea, CA, USA). Flow analysis was done to determine the proportion of migrating cells that displayed a phenotype indicative of progenitor cells.

### 2.3 Western Blots

BMSCs were treated with SFM (DMEM low glucose), 30 ng/mL BMP-2, 0.1 uM FTY720 or both for one hour. Then, samples were put on ice for 10 min, followed by centrifugation at 5000 rpm for 3 min. The supernatant was removed. Cells were lysed in a lysis buffer (Santa Cruz Biotechnology, Dallas, TX, USA) for 30 min, centrifuged at 4°C at 10,000 rpg for 10 min, and the supernatant was collected and run on a 4% acrylamide gel (Biorad, Hercules, CA, USA) for 30 min at 70 V and then 2 hours at 110 V. Proteins were transferred to a 45 um nitrocellulose membrane (Biorad). Finally, the membrane was blocked with 5% BSA (Santa Cruz Biotechnology) for 40 min on a shaker, then washed in 1× Tris buffered saline. The membrane was probed for either total smad-1 protein using anti-smad-1 antibody (Abcam, Cambridge, MA, USA) or phosphorylated smad-1 protein using phosphor smad-1 (ser206) mAB (Cell Signaling Technology, Danvers, MA, USA) and phosphor smad-1 (ser463/465) mAB (Cell Signaling Technology). Actin was used as a loading control. Protein was visualized using AlexaFLuor 680 labeled IgG (Invitrogen Life Technologies). Blots were imaged and quantified using a LiCor Odyssey (Licor Biosciences, Lincoln, NE, USA).

### 2.4 Differentiation Assay and Alizarin Red Staining

OP-9 cells, used to represent murine stromal cells, were cultured in osteogenic differentiation media composed of 10% FBS, 6 mM L-glutamine, 100 nM dexamethasone, 10 mM β-glycerol phosphate, 50 ug/ml L-ascorbic acid-2-phosphate and 1% penicillin/streptomyocin in DMEM for fourteen days. Additionally, cells were treated with 30 ng/ml BMP-2, 0.1 uM FTY720 in 3% FBS, or both compounds, in differentiation media. After fourteen days, cells were fixed with 10% formalin and stained with Alizarin Red (Sigma Aldrich, St. Louis, MO, USA).

The article "Delivery of Bioactive Lipids from Composite Microgel-Microsphere Injectable Scaffolds Enhances Stem Cell Recruitment and Skeletal Repair" was published in 2014. Journal: PLoS One.

### 2.5 qPCR

OP-9 cells were cultured in growth media and treated with 0.1 µM FTY720, 30 ng/ml BMP-2 or both for two weeks. RNA was harvested from the cells using the PureLink RNA kit, and reverse transcription was performed using a cDNA reverse transcription kit (Life Technologies). cDNA samples were diluted 1∶2 in water, and PCR was performed using primers for Runx2 with GAPDH as the internal control (Origene, Rockville, MD, USA). Real-time PCR was performed using the StepOnePlus system (Applied Biosystems, Carlsbad, CA, USA).

### 2.6 Synthesis of PLAGA microspheres

50∶50 poly(lactic-co-glycolic acid) (PLAGA) (5050DLF 5E, M_w_  = 65 kDa) (Lakeshore Biomaterials, Birmingham, AL, USA) were used to make microspheres encapsulating FTY720 (Cayman Chemical). Other solvents include methanol and methylene chloride (MeCl_2_) (Fisher Scientific, Pittsburgh, PA, USA), dimethyl formamide (Avantor Performance Materials, Center Valley, PA, USA), and poly (vinyl alcohol (PVA) and formic acid (Sigma Aldrich), and were used as received.

The single emulsion method was used to make FTY720-loaded microspheres. Briefly, FTY720 and PLAGA (1∶200 mass ratio) were dissolved in MeCl2 by sonication, with the resulting solution being 20% polymer (w/w). The organic solution was then slowly ejected into a 1% aqueous PVA (w/v) solution under stirring at 500 rpm overnight. The microspheres were collected by filtration, and dried under reduced pressure for 24 hours. Only microspheres with diameters of 50–300 µm were used for the study. Unloaded PLAGA microspheres were prepared similarly, but without the addition of FTY720. Scanning electron microscope (SEM) images of FTY720-loaded 50∶50 microspheres were taken.

### 2.7 In vitro Release of FTY720 from PLAGA Microspheres

FTY720 released from drug-loaded PLAGA microspheres was measured by extracting sphingolipid from the solution, and quantified via HPLC-MS. To measure extraction efficiency, either sintered microsphere discs or un-fused microspheres were placed in vials containing 1 mL simulated body fluid (pH 7.2; 7.996 g NaCl, 0.35 g NaHCO3, 0.3 g KCl, 0.136 g KH2PO4, 0.095 g MgCl2, 0.278 g CaCl2, 0.06 g MgSO4 in 1 L deionized water) with 4% (w:v) fatty acid free bovine serum albumin (FAF-BSA) and maintained at 37°C. The microspheres were moved to a new vial with fresh solution at each time point. A D-erythro-Sphingosine (C-17 base) internal standard was added (10 µL, 1 µM, Mw = 285.47 Da; Avanti Polar Lipids, Alabaster, AL, USA) to each sample. This mixture was sonicated for 15 min and immediately incubated at 48°C for 16 h. After cooling to room temperature, KOH (0.2 mL, 1 M) was added and the solution was centrifuged at 10,000 g for 10 min at 4°C. The supernatant was collected, dried to a solid with nitrogen air-flow and stored at −20°C. Immediately prior to HPLC-MS analysis, the extraction residue was dissolved in methanol (0.3 mL) and centrifuged at 12,000 g for 12 min at 4°C. Samples were analyzed with a Shimadzu UFLC High Performance Liquid Chromatograph (Shimadzu, Columbia, MD, USA) equipped with a Supelco Discovery C18, 5 µm (125 Å∼2 mm) connected to an ABI 4000 QTrap triple quadrupole mass spectrometer (Applied Biosystems).

The article "Delivery of Bioactive Lipids from Composite Microgel-Microsphere Injectable Scaffolds Enhances Stem Cell Recruitment and Skeletal Repair" was published in 2014. Journal: PLoS One.

### 2.8 Synthesis of Chitosan Gel

Chitosan from crab shells (minimum 85% deacetylation) (Sigma Aldrich) was dissolved in 0.5% acetic acid solution under magnetic stirring for 48 hours at room temperature. The resulting solution (pH −5.6) was filtered and stored at 4°C. 5 ml chitosan aliquot was taken in a glass vial and magnetically stirred in an ice bath. 60% ammonium hydrogen phosphate (AHP) solution in water at a pH −8.6 (Sigma Aldrich, St. Louis, MO) was slowly added to the chilled chitosan solution to form the gel.

### 2.9 Animal Defect Model

This study was carried out in strict accordance with the recommendations in the Guide for the Care and Use of Laboratory Animals of the National Institutes of Health. The protocol was approved by the University of Virginia Animal Care and Use Committee (Protocol Number = 3952). All surgery was performed under ketamine/xylazine anesthesia, and all efforts were made to minimize suffering. Sprague Dawley rats (280–300 grams in weight) were obtained from Charles River Laboratories International, Inc. (Wilmington MA, USA). Anesthesia was induced with isoflurane gas and continued with Ketamine/Xylazine (80/8 mg/kg IP). Following anesthetization, surgery was performed as described in Huang *et.al*. [18] in the laboratory during the morning hours. Briefly, after sterilization, a longitudinal incision was made through skin and periosteum, over the dorsum of the skull. The periosteum was reflected laterally. A 3 mm round burr was used to create an 8 mm defect in the bone with constant saline irrigation. The defects were treated with different scaffolds depending on the study. In all cases, the periosteum was closed with a 5–0 running nylon suture. The skin was closed with a running subcuticular vicryl suture, and VetClose (Butler Animal Health Supply, Dublin, OH, USA) was applied on the incision. Ketoprofen (3 mg/kg SC) was given after closure and for three days post surgery to minimize pain. Baytril (13 mL/bottle) was given orally via drinking water for a week following the surgery. Rats were housed according to ACUC guidelines, given free access to food and water and monitored for complications or abnormalities. The surgery procedure and postoperative care have been established in prior literature. At 9 weeks post-surgery, rats were anesthetized with 2.5% isoflurane gas and euthanized via cardiac injection with 1 mL Nembutal.

The article "Delivery of Bioactive Lipids from Composite Microgel-Microsphere Injectable Scaffolds Enhances Stem Cell Recruitment and Skeletal Repair" was published in 2014. Journal: PLoS One.

### 2.10 Treatments

Female Sprague Dawley rats (28) aged 8–10 weeks were assigned randomly to five different groups (n = 5–6). The animals were given one of the following five treatments: Only chitosan (C), chitosan with BMP-2 (2 µg) (CB), chitosan with PLAGA microspheres (M), chitosan with FTY720 in PLAGA microspheres (MF) (1∶200, drug: polymer) and chitosan with BMP-2+ FTY720 in PLAGA microspheres (BF).

### 2.11 MicroCT Measurement of Bone Growth

MicroCT of the defect regions was done at weeks 2, 4, 6 and 9 for all animals under ketamine/xylazine induced anesthesia using a VivaCT40 scanner (SCANCO Medical, Brüttisellen, Switzerland). 2D images were segmented by drawing the region of interest to comprise only parietal bone, which included all bone inside the ridges separating parietal from temporal bone. Animals were scanned with the following parameters: 38 µm voxel size, 55 kVp, 145 µA, medium resolution, 38.9 mm diameter field of view, and 200 ms integration time (73 mGy radiation per scan). Slice number was set for each animal throughout the study to include the whole defect and an equal length both anterior and posterior of the defect (≈300 slices). Bone was thresholded at 470.1–1000 mg hydroxyapatite (HA)/cm^3^, and bone volume was measured with the microCT software. 3D volume renderings were either done with SCANCO software after segmentation, or OsiriX 3.9 (Pixmeo, Geneva, Switzerland) from DICOM files of the region of interest. OsiriX images were thresholded and colored appropriately with the 16 bit color look up table (CLUT).

### 2.12 Microfil Enhanced MicroCT Measurement of Vascularization

After 9 weeks all cranial blood vessels were perfused with a contrast agent (Microfil) MV-122 (Flow Tech Inc., Carver, MA, USA), imaged and quantified with microCT. Rats were euthanized, the heart was exposed, and the common carotid arteries were cannulated, as performed previously [18]. Briefly, the arteries were ligated below the cannulation points, allowing direct perfusion of the vasculature in the neck and head region with 10 mL 2% heparin-saline from both sides. Then 3 mL Microfil mixed 1∶1 with diluent was perfused from each side over 5 min. The solution was allowed to set for 16 hours at 4°C. The calvarial sample including the defect and the surrounding parietal bone was harvested, fixated, decalcified and scanned in air with the following parameters: 21 µm voxel size, 45 kVp, 177 µA, medium resolution, 21.5 mm diameter field of view, and 200 ms integration time. Blood vessels in decalcified tissue were thresholded from 172–1500 mg HA/cm^3^, and the total blood vessel volume was quantified within an 8×9 mm^2^ area centered at the defect using Scanco software. Total vessel volume within the region of interest (ROI) was measured, and the total ROI size was kept constant for all evaluations. The volume occupied by vessels was determined by processing the raw image in ImageJ and Matlab to threshold vessel from surrounding tissue using a binary function.

The article "Delivery of Bioactive Lipids from Composite Microgel-Microsphere Injectable Scaffolds Enhances Stem Cell Recruitment and Skeletal Repair" was published in 2014. Journal: PLoS One.

### 2.13 Histology and Immunohistochemistry

Nine weeks after the initiation of treatment and after microCT evaluation, the animals were sacrificed and the calvarial bone was harvested for histological analysis. Briefly, the samples were fixed in 10% buffered formalin for 7 days and decalcified using an HCl and EDTA decalcifying solution (Richard-Allan Scientific, Kalamazoo, MI, USA) for 3 days at 4°C. The parietal bone was stored in 70% ethanol until paraffin embedding for staining with Mason's Trichrome and Hematoxylin and Eosin. Paraffin sections were de-waxed, permeabilized with 0.1% Triton X-100, and blocked for 2 hours with 1% donkey serum and 1% goat serum. Sections were immunolabeled for 16 hours at 4°C with a monoclonal CD45 murine antibody (Santa Cruz Biotechnology) diluted 1∶100 in (PBS, 0.1% saponin, 0.1% BSA) a CD90 murine antibody (Biolegend) or a polyclonal CD29 rabbit antibody (Novus Biologicals, San Diego, CA, USA) both diluted 1∶400 in PBS. After washing 3× in PBS, the sections were incubated for 1 hour at room temperature with donkey anti-mouse AlexaFluor 488 (Abcam) and/or goat anti-rabbit AlexaFluor 568 (Molecular Probes) secondary antibodies, both diluted 1∶200 in PBS. Labeled sections were then washed and mounted with 100 mM glycine in PBS. Sections were imaged on a Zeiss LSM 700 confocal microscope (Zeiss, Thornwood, NY, USA).

### 2.14 Statistical analysis

Results are presented as mean ± SEM. Statistical analysis of the increase in bone and blood vessel volume was performed using ANOVA, followed by post hoc Tukey's Test for pair-wise comparison. Grubb's test was used for outlier analysis. For all histological analysis, the defect region was divided into 2 regions and 3 consecutive slices from each animal were used for quantification.

## Results

### 3.1 FTY720 enhances migration and differentiation of osteoblast precursors towards SDF-1

SDF-1 is increased in the periosteum of injured bone [24] and enhances the recruitment of osteogenic cells from the peripheral circulation to the site of bone repair [25]. Transwell migration assays conducted on whole bone marrow pretreated with BMP-2, FTY720 or their combination were used to assess the effect of these factors on cell migration via SDF-1 and S1P dependent pathways (***Figure 1a–c***). This whole marrow migration assay enables the assessment of effects of BMP-2, FTY720, or both on the migration capability of different cells while maintaining the microenvironment of the bone marrow. We see that FTY720 pre-treatment of whole bone marrow cells increases their migration towards SDF-1, but not S1P, (compared to serum-free media) suggesting that FTY720 activation of S1P receptors 1 and 3 stimulates the SDF-1/CXCR4 axis (Figure 1b). Furthermore, we see increased transmigration of bone marrow stromal cells overall, both in the presence and absence of an SDF-1 or S1P chemokine gradient stimulation, suggesting that cells exposed to the combination of FTY720 and BMP-2 exhibit greater motility (chemokinesis) (***Figure 1c***). Among those cells that migrate across the transwell membrane from the marrow stoma, subsequent flow cytometry analysis reveals a significant increase in SDF-1 mediated chemotaxis by CD90+/CD45-/CD11b- cells (a phenotype indicative of MSCs) (***Figure 1d***). Western blot analysis (***Figure 2a***) shows that smad-1 phosphorylation in BMSCs increases when treated with FTY720 compared to BMP-2. Flow cytometry analysis after treatment of CD90+/CD29+/Sca1+ murine MSC cells also showed that treatment with FTY720 enhanced BMP-2 induced smad-1 activity (as measured by phospho-smad-1 events) (***Figure 2b–c***). This increase in smad-1 phosphorylation is consistent with the transwell migration results, implying that smad-1 could be involved in enhancing progenitor cell migration following FTY720 stimulation. Additionally, FTY720 treatment also enhances the mineralization of progenitor cells like OP-9 cells as shown by Alizarin red staining (***Figure 2d***). This is also consistent with an increase in the mRNA expression of the Runx2 gene that is differentially expressed in the early stages of osteoblastic differentiation (***Figure 2e***).

The article "Delivery of Bioactive Lipids from Composite Microgel-Microsphere Injectable Scaffolds Enhances Stem Cell Recruitment and Skeletal Repair" was published in 2014. Journal: PLoS One.

**Figure 1:** FTY720 increases progenitor cell migration and differentiation. (A) Schematic of transwell assays used to measure the migratory ability of BMSCs pre-treated with FTY720, BMP-2, both or neither towards, serum free media, SDF-1 or S1P. (B) Treatment with FTY720 increases chemotaxis towards SDF-1. (C) Addition of FTY720 to BMP-2 treatment enhances cell motility. (D) Treatment with FTY720 increases SDF-1 mediated chemotaxis of CD90+ cells, as measured by flow cytometry, normalized to SFM. (** p<0.01 & *p<0.05)

**Figure 2:** FTY720 increases smad-1 mediated osteogenic differentiation of progenitor cells. (A) Western blot analysis of BMSCs reveals increase in smad-1 phosphorylation when treated with FTY720 compared to BMP-2. (B–C) Flow cytometry for phosphor-smad in murine MSCs reveals FTY720 treatment enhances BMP-2 induced smad-1 activity. (D) FTY720 enhances mineralization of progenitor cells, shown by Alizarin Red and (E) qPCR shows increase in Runx2 mRNA in progenitor cells when treated with FTY720, shown as fold change over SFM. (** p<0.01 & *p<0.05).

### 3.2 In vitro release of FTY720 from 50∶50 PLAGA microspheres is sustained over 4 weeks

We explored the development of 50∶50 PLAGA microsphere formulations for delivery to CSDs encapsulated within injectable chitosan microgels. ***Figure 3a*** shows SEM images of these microspheres loaded with FTY720 (1∶200 drug to polymer ratio) as well as the *in vitro* release of FTY720 from PLAGA microspheres into simulated body fluid, which was measured over a period of 4 weeks to ensure sustained release of the molecule from PLAGA. The encapsulation efficiency of FTY720 in the microspheres was 70%, as measured by LC-MS. Despite the relatively small size of the FTY720 molecule, we observed continuous release of the drug over a 4 week period of *in vitro* evaluation. The release over the first week is approximately linear, with an increasing rate of release between weeks 2 and 4. The latter may suggest a drug release aided by polymer degradation. This *in vitro* release data implies that FTY720 is actively released from the microspheres even after 4 weeks of implantation [26], [27]. This may be attributed to possible hydrophobic interactions between FTY720 and PLAGA that causes a slower release rate over a period of weeks as previously reported [28]. This interaction could be beneficial for tissue engineering applications such as bone regeneration as the therapeutic effect of FTY720 would be sustained over a longer period of time. The schematic for the *in vivo* experimental hypothesis is outlined in ***Figure 3b***.

**Figure 3:** FTY720 is released from PLAGA microspheres over 28 days. (A) Fraction of FTY720 release from PLAGA microspheres with a drug to polymer ratio of 1∶200. The encapsulation efficiency in the microspheres was 70%. Inset: SEM micrograph of FTY720-loaded PLAGA microspheres (scale bar  = 100 um). (B) Schematic of in vivo experimental hypothesis.

### 3.3 FTY720 accelerated bone growth in rat CSDs

CSDs in rats were treated with FTY720 loaded 50∶50 microspheres delivered in a chitosan gel with or without BMP-2. Since the rate of bone growth is critical for healing, cumulative new bone formation was assessed for all animals at weeks 2, 4, 6 and 9 using microCT. ***Figure 4a-d*** shows the cumulative bone growth in the defect regions over this period for all the different treatment conditions normalized to the vehicle (chitosan only) group. The group treated with FTY720- PLAGA microspheres shows a higher amount of bone growth in the defect region, as early as 2 weeks post treatment. Histological evaluation of cranial sections at 9 weeks stained with Masson's trichrome is shown in ***Figures 5a–e***. H&E and Masson's trichrome staining show that the number of osteoblasts and the quantity of osteoid tissue in the defect regions was greater in groups treated with FTY720 (***Figures 5*** ***&*** ***6***).

The article "Delivery of Bioactive Lipids from Composite Microgel-Microsphere Injectable Scaffolds Enhances Stem Cell Recruitment and Skeletal Repair" was published in 2014. Journal: PLoS One.

**Figure 4:** Bone growth in the critical size cranial defect measured using microCT. The ratio of bone volume (BV) to total volume (TV) of the region analyzed by microCT indicates the cumulative amount of new bone formed at (A) Week 2, (B) Week 4, (C) Week 6 and (D) Week 9 after implantation (** p<0.01 & *p<0.05 compared to chitosan control; αα p<0.01 & α p<0.05 compared to PLAGA control at similar time points). Representative images of a quadrant of the defect site are shown at each time point (White dashed lines indicate original defect, white arrows indicate new bone formation.

**Figure 5:** Masson's trichrome stain for bone growth in cranial defect at week 9 after treatment with (A) Chitosan, (B) Chitosan + PLAGA microspheres, (C) Chitosan + PLAGA microspheres loaded with FTY720, (D) Chitosan loaded with BMP-2 and (E) Chitosan loaded with BMP-2 + PLAGA microspheres loaded with FTY720. In the FTY720 groups there is increased bone formation in the defect void space compared to the BMP-2 group and vehicle controls. FTY720 treatment results in the formation of light osteoid bodies (asterisk) and mature bone (arrowhead) (scale bar  = 1 mm).

**Figure 6:** FTY720 enhances osteoblast number and reduces inflammatory cell recruitment in the defect region 9 weeks after injury. (A) Chitosan, (B) Chitosan + PLAGA microspheres, (C) Chitosan + PLAGA microspheres loaded with FTY720, (D) Chitosan loaded with BMP-2 and (E) Chitosan loaded with BMP-2 + PLAGA microspheres loaded with FTY720. Top row: Number of osteoblasts increases in the defect region after treatment with FTY720 (scale bar  = 100 um). The average number of osteoblasts after H&E staining is determined by counting cells around newly formed osteoid regions (black arrows). Representative H&E stain for bone growth in cranial defect at week 9 afterFTY720 treatment results in the formation of more osteoid regions in the defect area (white arrow). This is quantified from images taken from the center of the defect region (F) (*p<0.05 compared to chitosan control; ^α^ p<0.05 compared to PLAGA control). Middle row: FTY720 treatment reduces CD45+ inflammatory cells in defect (scale bar  = 500 um). Bottom row: FTY720 treatment leads to enhanced recruitment of CD90+/CD29+ cells to the defect site (white arrows indicate co localization).

The article "Delivery of Bioactive Lipids from Composite Microgel-Microsphere Injectable Scaffolds Enhances Stem Cell Recruitment and Skeletal Repair" was published in 2014. Journal: PLoS One.

As it is possible that newly mineralized bone fell below the microCT detection threshold, we used high magnification of the H&E staining (***Figure 6*** ***, top row***) to identify osteoblasts around newly formed osteoid regions (indicated with black arrows). FTY720 treated groups show more mature bone (white arrows) in the defect region along with the formation of new osteoid bodies. The number of osteoblasts, counted in the center of the defect region, is higher for the groups that were treated with FTY720, resulting in increased bone growth in the defect region. Immunofluorescence staining at 9 weeks post-injury revealed lower CD45 staining in groups treated with FTY720, suggesting a potential immunomodulatory effect (***Figure 6*** ***, middle row***), which could lead to increased transport of osteogenic precursors or supportive cells to the defect site. To determine progenitor cell recruitment to the defect area in response to local FTY720 treatment, cranial defect sections were co-stained for both CD29 (red) and CD90 (green) (***Figure 6*** ***, bottom row***), which are markers of mesenchymal stem cells [27]. The two markers displayed high co-localization (amber) indicating presence of MSCs (white arrows). The FTY720 treated groups showed higher numbers of CD29+CD90+ cells than the BMP-2 only treated group, and even less in the chitosan and PLAGA microsphere groups. This finding suggests that local FTY720 treatment enhances the recruitment of MSCs towards injury sites, supporting the *in vitro* findings described previously.

### 3.4 FTY720 enhanced defect site vascularization in rat CSDs

Vascularization is crucial to bone defect healing, as microvessels accelerate bone formation even before blood flow has been established [29]. Following inflammation modulation, osteoblast precursors [30] and support cells such as potentially osteogenic pericytes [31] travel through the vasculature to reach the injury site. Additionally, blood vessels have been shown to serve as a scaffold for osteoblast differentiation [32], [33]. ***Figure 7b–f*** shows representative microCT images of Microfil-enhanced vasculature of the defect site 9 weeks after treatment with the different therapies. The number of mature vessels is substantially higher after FTY720 treatment and this difference is maintained even after 9 weeks. The area occupied by the blood vessels in the defect region is quantified in ***Figure 7a***. This result suggests that increased vascularization could play a critical role in accelerating the increased bone growth observed with FTY720 treatment.

The article "Delivery of Bioactive Lipids from Composite Microgel-Microsphere Injectable Scaffolds Enhances Stem Cell Recruitment and Skeletal Repair" was published in 2014. Journal: PLoS One.

**Figure 7:** FTY720 enhances vascularization in a critical size cranial defect. (A) Vascularization in the critical size cranial defect measured using microfil enhanced microCT imaging. (B–F) Volume in the defect region occupied by vessel ingrowth 9 weeks after different treatments (** p<0.01 & *p<0.05 compared to chitosan control; αα p<0.01 & α p<0.05 compared to PLAGA control) MicroCT images showing vessel and bone in-growth at week 9 for animals treated with (B) Chitosan, (C) Chitosan + PLAGA microspheres, (D) Chitosan + PLAGA microspheres loaded with FTY720, (E) Chitosan loaded with BMP-2 and (F) Chitosan loaded with BMP-2 + PLAGA microspheres loaded with FTY720.

## Discussion

Recent reports of complications such as graft failure, infections and unwanted bone formation after BMP-2 usage highlights the need for alternative therapies [34]. The development of strategies that harness the recruitment of endogenous bone progenitor cells and enhance defect site vascularization may be effective at augmenting the local effects of osteoinductive molecules such as BMP-2. Our lab has previously shown that local delivery of FTY720 promotes local arteriogenesis and allograft integration in a rat cranial defect model [16], [17], [18]. Additionally, we have shown that FTY720 release from hard tissue scaffolds enhances osseous integration, accelerates vascularization across the host-graft interface, resolves chronic inflammation, and directs anti-inflammatory cell recruitment [17], [18], [22], [28]. In this study, we explore a biomaterial-based delivery platform of FTY720 for modulation of a host of processes critical in bone repair, including inflammatory response, vascularization, and recruitment of endogenous bone progenitor cells.

While our material of choice, chitosan, has been used for various tissue-engineering applications such as healing of myocardial infarcts, bone regeneration and cartilage renewal [2], [35], [36], recent studies have shown that chitosan as a scaffold can enhance mineralization during osteoblast differentiation [37]. Although chitosan alone does not result in substantial defect healing [2], [38], use of such an injectable biomaterial is clinically relevant for craniofacial surgery where using an injectable therapeutic platforms can be beneficial due to ease of application. As FTY720 is a hydrophobic drug, it is ideal for incorporation into hydrophobic PLAGA microspheres in order to achieve sustained delivery. Though release kinetics of FTY720 from such microcarriers differs from pure diffusion out of a gel, we have shown in prior studies that the microsphere/microgel formulation positively impacts the pattern of bone growth [39]. Due to the fact that microspheres made of 50∶50 PLAGA swell and lose their architecture relatively quickly when delivered on their own *in vivo*, suspension of these microcarriers within chitosan imparts sustained release kinetics of FTY720 over 4 weeks [39]. Stephan et al. previously showed that delivery of mesenchymal stem cells along with BMP-2 in an injectable scaffold increases bone formation over either therapeutic alone [2]. Here, we investigate the replacement of exogenous cell delivery with a small-molecule, FTY720, capable of recruiting endogenous progenitor cells. Our results suggest that optimizing injectable scaffolds dually delivering FTY720 and BMP-2 could potentially result in a cell free therapy for CSDs in cranial bone.

The article "Delivery of Bioactive Lipids from Composite Microgel-Microsphere Injectable Scaffolds Enhances Stem Cell Recruitment and Skeletal Repair" was published in 2014. Journal: PLoS One.

The results of FTY20 delivery in chitosan microgels are consistent with previously reported *in vivo* findings. Delivery of FTY720 promotes the development of a vascular network in the vicinity of a cranial defect that may enable the recruitment and differentiation of bone progenitor cells due to increased blood flow and growth factor/nutrient delivery. Locally delivered FTY720 has been shown to result in an increase in vascular length and density [40], [41]. Microfil enhanced microCT in our CSD study similarily showed that local FTY720 treatment resulted in enhanced vascularization of the defect region, a phenomenon that persisted 9 weeks post-injury (***Figure 7***). Though approaches involving local delivery of VEGF to increase blood supply around a bone fracture site have been shown to increase healing [40], signaling through S1P receptors not only stimulates endothelial morphogenic processes, such as lumen formation and branching [42], [43], but also promotes mural cell recruitment, (mediated through S1P receptor subtype 1 (S1P_1_)), resulting in more stable vasculature at the defect site.

We report for the first time how potential signaling crosstalk between S1P receptors (S1PRs), chemokines, and growth factors that are active during bone wound healing may substantially enhance bone progenitor recruitment. It is well known that SDF-1 production increases at the site of injury [24] and SDF-1/CXCR4 signaling plays a significant role in the initiation of MSC differentiation and declines once the cells choose a differentiation pathway [44], [45], [46]. Thus, we were particularly interested in whether crosstalk between S1P receptor activation via FTY720 and the endogenously active SDF-1/CXCR4 axis in the healing microenvironment may enhance migration of progenitor cells toward injected chitosan microgels. Our results provide evidence that bone marrow derived cells exhibit enhanced chemotaxis towards SDF-1 after pre-treatment with FTY720 (***Figure 1b***). When we perform flow cytometry analysis on the migrated cells, we found that the population of cells that displayed enhanced chemotaxis was enriched for the CD90+/CD11b-/CD45- phenotype (***Figure 1c***), one that is indicative of mesenchymal stem cells. Therefore, locally delivering FTY720 at a site of bone injury may enhance endogenous progenitor cell migration via synergistic effects of S1P receptor activation of SDF-1/CXCR4 signaling.

The article "Delivery of Bioactive Lipids from Composite Microgel-Microsphere Injectable Scaffolds Enhances Stem Cell Recruitment and Skeletal Repair" was published in 2014. Journal: PLoS One.

Though the dual treatment of BMP-2 and FTY720 did not yield substantially better results than treatment with FTY720 alone, many factors must be considered. It is possible that a longer study is required to tease out the impact of the dual treatment compared to each factor alone, as FTY720 and BMP-2 may act in bone wound healing on different time scales. The second issue is that of dosage. Higher doses of BMP-2 have been shown to have substantial impact on bone regeneration, though too high a dose has led to negative consequences. We chose a BMP-2 dosage (2 µg) comparable to that published by Stephan *et.al*. in an effort to compare two strategies that increase mesenchymal stem cell number at the defect site [2]. However, it is possible that titrating the dose of BMP-2 for delivery beside a recruitment factor vs. exogenous cells is required in order to achieve comparable bone growth.

Though complete healing in the cranial defect was not observed, significantly higher bone formation was measured at the defect site in the FTY720 treated animals compared to those treated with BMP-2. The surprising effectiveness of FTY720 may be attributed to the underlying effects on bone progenitor recruitment. Previous studies have shown that FTY720 promotes SDF-1/CXCR4 dependent migration of hematopoietic stem cells into the bone marrow in a S1P_1_ dependent manner [47] and the osteoblastic differentiation of C2C12 cells [48]. Though S1P_2_ activation in pre-osteoblasts serve as a chemo-repellant receptor [38], FTY720 has no activity at S1P_2_, thus its role in the bone healing environment would not hinder pre-osteoblast migration to the site of injury. In addition, we've shown that activation of S1P_3_ signaling results in a concentration dependent phosphorylation of smad-1 and smad-2 proteins, members of the smad family of intracellular signaling molecules (***Figure 1d-e*** **)**. Smad-1 is known to transduce signals from BMP-2 receptors, indicating the cross activation of this signaling pathway by S1P_3_ activation [49]. Additionally, activation of S1P_3_ has also been shown to activate CXCR4 signaling [50], which can also contribute to the observed increased recruitment of MSCs to the injury site (***Figure 6***). Future studies will be required to determine the respective contributions of enhanced chemokinesis and directed SDF-1 mediated chemotaxis among cells treated by the combination of the two factors.

The article "Delivery of Bioactive Lipids from Composite Microgel-Microsphere Injectable Scaffolds Enhances Stem Cell Recruitment and Skeletal Repair" was published in 2014. Journal: PLoS One.

The inflammatory response at the injury site is also a critical determinant of the rate of regeneration [43], [51]. While inflammation initiates the various steps of healing, uncontrolled up-regulation of pro-inflammatory cytokines could negatively impact the process of regeneration [52]. Local suppression of inflammation has also been shown to increase the effect of BMP-2 in critical size defect healing [53]. FTY720 has been shown to suppress inflammation when delivered both locally [54] and systemically [55]. S1P receptor activation is also known to play an important role in myeloid cell recruitment during acute inflammation [56] and promote the recruitment of monocytes and macrophages in atherosclerosis [57]. We've recently shown that local delivery of FTY720 can tune the local inflammatory environment in a manner that may be beneficial to processes involved in bone regeneration, such as arteriogenesis, by selectively recruiting anti-inflammatory monocytes, and skewing the local cytokine profile towards a more pro-regenerative milieu [22]. Similarly, we've shown in a previous study that local delivery FTY720 to a mandibular defect promotes recruitment of alternatively-activated, pro-regenerative “M2” macrophages 3 weeks post-injury [28]. It is possible that local delivery of FTY720 in a cranial defect also harnesses local inflammation in a similar manner to promote bone formation, though these effects may manifest at earlier time points than the ones investigated here. In this study, we looked at CD45+ cells in the defect area 9 weeks post-injury, and observed a decrease in CD45+ cells with FTY720 treatment, suggesting an attenuation of any persisting inflammation at the defect site. Further studies at earlier time points are required to determine the shorter-term role of FTY720 on inflammation in regenerating bone.

## Conclusions

In summary, this study explored the potential use of appropriately engineered signaling lipid biomolecules for promotion of endogenous bone repair. This study shows that local delivery of a selective S1P receptor agonist can be used to increase bone growth in the initial weeks following traumatic injury, in addition to modulating local inflammation and enhancing migration of endogenous bone progenitor cells. The injectable composite microsphere/microgel formulation used here is a promising drug delivery platform that represents a viable alternative to cell-based therapies via recruitment of endogenous progenitor cells.
